RETRACTED

# Delayed Surgery to Preserve Kidney with Grade IV Injury

**DOI:** 10.1155/2022/5066278

**Published:** 2022-09-22

**Authors:** YunPeng Li, Long Xiao, WanChao Xu, Liangyun Zhao, MinHui Xiao

**Affiliations:** ^1^Department of Urology, The Fourth People's Hospital of Yunnan Province, Dali 671000, China; ^2^Department of Urology, Yunnan First People's Hospital, Kunming 650000, China

## Abstract

**Background:**

Since the introduction of the ALARA (“as low as reasonably achievable”) concept, the management of severe renal trauma has shifted. Our hospital promotes delayed surgical intervention for grade IV closed renal injury, to preserve renal function. In this study, we retrospectively reviewed the management and outcomes of patients with grade IV closed renal injury in our hospital.

**Objective:**

To evaluate the management and outcome of grade IV closed renal injury.

**Methods:**

We retrospectively reviewed the medical records of 45 patients with grade IV closed renal injury; namely, 36 men and 9 women with an average age of 35.6 years. All patients were diagnosed with grade IV closed renal injury in accordance with the guidelines of the American Association for the Surgery of Trauma. All hemodynamically-stable patients with renal trauma were treated conservatively for approximately 13 days and then underwent surgery only to clear the perirenal hematoma and not to repair or resect the affected kidney. Abstracted data included patient demographics, mechanism of injury, admission hemodynamics, CT findings, and mortality. The primary outcome was the success rate of nonsurgical treatment, and the secondary outcome was the complication of nonsurgical treatment.

**Results:**

All patients responded and were discharged, and no patients died. We followed 35 (77.8%) patients for at least 1 year. One patient with partially devitalized renal parenchyma underwent surgery to remove the affected kidney. Eleven patients (31.4%) suffered complications, namely, three (8.6%) cases of hypertension, four (11.4%) cases of hematuria, two cases (5.7%) of urinary tract infection, and two (5.7%) cases of urinoma.

**Conclusions:**

Delayed exploratory surgery only to remove the hematoma should be considered in hemodynamically-stable patients with grade IV closed renal injury. This approach can avoid high nephrectomy rates associated with emergency surgery and reduce the complications that result from conservative treatment without surgery.

## 1. Introduction

Traumatic kidney injury accounts for about 5% of all surgical injuries and is a common urological emergency. Kidney trauma is most common in traffic accidents, falling from a high altitude, and sports injuries [1–3]. Most of the local renal injury was low blunt renal injury (grades I–III), and others were severe renal injuries. Low-grade blunt kidney injury can be resolved by conservative treatment, which is widely accepted. However, severe renal injury, including grade IV and V blunt renal injury (renal fragmentation, hilar vascular tear, dissection with no blood supply to the kidney), requires surgical intervention, and nephrectomy is considered to be the appropriate treatment [4]. Due to limited prospective studies, the treatment of grade IV blunt renal trauma is controversial and there is no optimal treatment strategy. In the emergency treatment of this level of renal injury, the report indicates that surgery is unavoidable and that nephrectomy is necessary due to the location of the injury and associated vascular damage [4]. A review study showed that emergency nephrectomy was more common than nephron-sparing surgery in patients with grade IV blunt renal trauma [2, 3]. Intraoperatively, urologists are often unable to repair damaged kidneys in patients with grade IV blunt renal trauma due to acute renal hemorrhage, inflammation, severe trauma, perirenal hematoma, or anatomical confusion, leading to nephrectomy [5, 6]. In other studies, some patients with grade IV blunt renal trauma received only conservative treatment, and CT showed renal laceration involving the renal cortex, medulla, and collecting system, injury involving the main arteries and veins of the kidney, and segmental renal infarction without renal laceration. In addition, for patients with stable hemodynamics, conservative treatment and observation are commonly used, and a series of imaging examinations are required due to the concomitant injury of other abdominal organs. Therefore, emergency surgical intervention is necessary, resulting in the removal of the affected kidney [7]. Based on these findings, management of grade IV blunt kidney injury remains an important clinical issue [8].

RETRACTED

In our institution, from February 1994 to March 2016, hemodynamically-stable patients with grade IV closed renal trauma underwent conservative treatment for approximately followed by surgery only to remove the perinephric hematoma. This approach increased the likelihood of nephron-sparing compared with emergency surgery, and also significantly decreased the long-term complication rate. We describe our findings in these patients, in this report.

## 2. Methods

### 2.1. General Information

This is a retrospective case series including all adult patients with a grade IV blunt renal injury who were admitted between February 1994 to March 2016, to a third-class hospital in Yunnan Province, China. Renal injuries were graded based on computed tomographic (CT) findings and according to the American Association for the Surgery of Trauma Organ Injury Scale [1] which was defined as laceration through the parenchyma into the collecting system, vascular segmental venous or arterial injury, and any injury involving the collecting system (renal pelvis laceration and ureteric kidney pelvic disruption).

Based on these criteria, 45 patients with grade IV blunt renal injuries were included. We excluded patients with hemodynamic instability, other mental disorders, cognitive disabilities, or severe dysfunction of the heart, liver, and lung; included patients consisting of 36 men and nine women, with an age range of 4–72 years and an average age of 36.5 years (as shown in Table 1). Twelve patients sustained collision-related trauma, 27 sustained injuries following traffic accidents, and six patients experienced falls. Of the 45 patients, 24 patients sustained right kidney injury, and 21 patients sustained left kidney injury (as shown in Table 2). Based on patients' clinical manifestations, lower back pain was the most common complaint; gross hematuria occurred in 33 patients, and microscopic hematuria occurred in 12 patients. Physical examination revealed tenderness, a local mass, and percussion pain at the trauma site most often; two patients presented with ecchymosis, 24 patients presented with fever, and two patients presented with severe fever (> 39°C).

## 3. Treatment Methods

Methods After admission, all patients underwent routine urine examination, ultrasound examination, and CT examination and were confirmed to have grade IV closed renal injury (Figure 1). Conservative treatment lasted for about 13 days. Specific measures were as follows: first, ensure successful hemostasis, ensure the amount of blood transfusion when necessary, and monitor the patient's vital signs; nursing staff considers continuous testing of hematocrit measurement, let the patient rest in bed; consider clinical monitoring of the patient's physical condition and administer iv fluids if necessary. Treated with “Huayu Zhuxue Decoction” of traditional Chinese medicine: 10 g of raw dandelion, 12 g of dandelion, 6 g of wulingzhi, 15 g of white peony, 12 g of red peony, 6 g of peach kernel, 12 g of *Angelica sinensis*, 15 g of Achyranthes bidentata, 9 g of Dipsacus, 6 g of Jing mustard, 6 g of Panax notoginseng powder (for flushing), 6 g of roasted licorice, 24 g of chenneijin, 24 g of haijinsha and 3 g of amber powder (for flushing); 1 dose per day. Patients underwent surgery only to remove the perirenal hematoma and not to repair the lacerated kidney (Figure 2). Intraoperatively, we removed the perirenal organizing hematoma and addressed any urine extravasation. We did not dissect and control bleeding from the renal artery, which increased the ease and safety of the surgery. As seen in Figure 2, the lacerated edges of the kidney adhered closely to each other and were well-restored because of the organizing hematoma, which eliminated the need for further renal repair or nephrectomy. More recently, we used a laparoscope to remove the perinephric hematoma in some patients, and also achieved satisfactory results. We use and recommend an indwelling perinephric drainage tube (Figure 3).

RETRACTED

## 4. Data and Outcomes

The following data were collected: demographics, mechanism of injury (collision-related trauma, traffic accidents, and fall), admission hemodynamics, CT findings, presence of free abdominal blood on CT scan (recorded as diffuse or confined around the kidney), and mortality. The primary outcome was the success rate of nonsurgical treatment, and the secondary outcome was the complication of nonsurgical treatment.

### 4.1. Statistical Analysis

SPSS 24.0 statistical software was used for analysis and statistical description according to data type. The measurement data conforming to normal distribution are expressed in mean ± standard deviation, the measurement data not conforming to normal distribution are expressed in median and quartile, and the counting data are expressed in frequency and percentage.

## 5. Results

All 45 included patients with grade IV closed renal injury underwent delayed surgical intervention, and one patient required nephrectomy secondary to poor adherence to the laceration margins. Kidneys in all remaining patients were successfully preserved, intraoperatively, and no patients died (as shown in Table 3).

Postoperative follow-up was performed for 35 patients for at least 1 year. Eleven of the 35 patients (31.4%, 11/35) developed complications related to kidney trauma(as shown in Table 2), namely, hypertension in three patients (8.6%, 3/35), for whom oral antihypertensive drugs controlled the symptom; four patients (11.4%, 4/35) developed microscopic hematuria; two patients (5.7%, 2/35) developed urinary tract infection, which responded to antibiotic therapy; and two patients (5.7%, 2/35) developed urinoma, which was treated with an indwelling drainage tube and which gradually dissolved (as shown in Table 4).

## 6. Discussion

Renal injury accounts for approximately 10% of all trauma cases, and the majority of patients sustain blunt renal trauma. The management of the renal injury is based on the mechanism of the injury, associated injuries, hemodynamic stability, and severity. Traditionally, grades I–III injuries have been managed conservatively, while patients with grade V injuries almost always undergo surgical exploration. For patients with severe renal injury (grades IV–V), except when life-saving measures are necessary; preserving renal function and minimizing the complications associated with kidney trauma should be the aim of therapies.

RETRACTED

According to the criteria for nomenclature and classification of acute kidney injury agreed by the Taiwan AKI Working Group in 2021, grade IV laceration kidney injury runs through the renal cortex, medulla, and collecting system, and damage in the main branches of renal arteries and veins accompanied by bleeding can be treated conservatively or repaired in an emergency or delayed manner according to the actual situation of patients [9, 10]. Sun reported [11] that, in a cohort of 22 patients with a renal injury who underwent surgical intervention, nephrectomy was performed in 59% of patients. Su et al. [12] reported that 12 patients with severe kidney injury underwent surgery, and a nephrectomy was performed on 10 patients. In hemodynamically-stable patients with severe blunt renal trauma, choosing whether to perform surgery or nonoperative management can be difficult. The treatment of grade IV injuries is even more controversial because these patients can be managed conservatively or undergo urgent repair or delayed repair. Currently, most clinicians choose conservative treatment to avoid unnecessary nephrectomy and other unexpected risks [13]. Van et al. [14] reported, in a multicenter study of the nonsurgical treatment of severe blunt renal trauma in hemodynamically-stable patients, that the failure rate of nonsurgical treatment was only 6.5%. In the study, there were two important predictors: one was patient age > 55 years, and the other was vehicular trauma. If patients with grade IV or V renal trauma had both of these predictors and received conservative treatment, the failure rate was as high as 27.3%. Furthermore, the inconvenience and complications of conservative management increased patients' difficulties. Long periods of bed rest were extremely difficult for patients, especially for vital and active young children [15, 16]. Moreover, perirenal hematoma, if not cleared in time, may lead to infection and abscess formation, possibly even tissue fibrosis, which leads to hydronephrosis and more difficult future management.

Among our patients prior to the current study, 2 years after renal injury, two patients receiving conservative treatment required nephrectomy because of refractory hypertension. Therefore, we adopted the delayed exploratory surgery approach to treat patients with severe closed renal injury (grade IV). Specifically, hemodynamically-stable patients currently undergo conservative treatment for approximately 13 days and then undergo exploratory surgery, only to remove the perirenal hematoma. This approach is possible because of the “self-healing” ability of the kidney, which eliminates the need for kidney repair and reduces the surgical risk and difficulty. During conservative treatment, we used plain CT to dynamically observe the affected kidney, which can correctly have evaluated the extent of renal injury, determine the scope of the urinary extravasation and hematoma, and reveal devitalized renal tissues. CT examination is an important diagnostic and monitoring tool when evaluating renal injury [17–20]. In this study, raw dandelion, wulingzhi, peach kernel, and Schizonepeta were used to activate blood circulation and remove blood stasis, and Danpi was used to induce various drugs to the kidney to remove blood stasis and heat; *Angelica sinensis* and pseudo ginseng can not only promote blood circulation and remove blood stasis but also stop bleeding. We chose delayed exploratory surgery for several reasons. First, the kidney has a rich blood supply and strong compensatory and repair capability, often self-repairing once bleeding stops (Figure 4). Second, because patients undergo approximately 13 days of conservative treatment, delaying surgery avoids active hemorrhage resulting from the initial renal trauma. Because there is no active hemorrhage during the delayed surgery, and the surgical view is clear, urologists can operate precisely and better protect the kidney. Third, during delayed exploratory surgery, renal tissue edema has almost disappeared, and no conspicuous tissue adhesions between the kidney and surrounding tissues are present. Urologists can then more easily dissect the perirenal tissue and reveal the renal wound. Thirteen days after injury, renal tissue repair has passed the inflammatory stage and entered the tissue proliferation and granulation stage. It is well-known that granulation tissue fills and repairs the renal tissue wound, and has a strong resistance to infection. Therefore, because granulation tissue is not removed, it can provide a physiological basis for patients' rehabilitation. Although postoperatively, complications such as urine extravasation, hypertension, urinary infection, and urinoma are possible, the incidence of these complications is significantly lower compared with conservative treatment without delayed surgery [6, 7] If exploratory surgery is performed early after injury (< 10 days), although the surgical approach is easier, renal wound healing is poor and often requires repair, which increases the surgical difficulty. In contrast, if the exploratory surgery is delayed too long, because of renal fat adhesion and tissue organization, it is more difficult to identify the kidney and renal wound. Therefore, we recommend appropriately-delayed surgical treatment for hemodynamically-stable patients with grade IV closed renal injury to avoid the high nephrectomy rates associated with emergency surgery and to reduce the complications that result from conservative treatment without surgery. Delayed surgical intervention was appropriate for patients with grade IV closed renal injury, in our study.

RETRACTED

## 7. Limitation

The study was subject to a number of limitations. First, because of the small number of patients, follow-up was difficult, and the lost-to-follow-up rate was high; no information on complications was available for the patients lost to follow-up. Second, because of the retrospective design and a lack of prospective information; therefore, data discrepancies were unavoidable.

## Figures and Tables

**Figure 1:** Computed tomographic image showing grade IV closed renal trauma. The perirenal hematoma is large and indicated by the arrow.

**Figure 2:** Intraoperative video image showing the perirenal organizational hematoma during the delayed surgery.

**Figure 3:** Computed tomographic image after the perirenal hematomas have been removed. The arrow indicates the perinephric drainage tube.

**Figure 4:** Intraoperative video image showing the self-healing ability of the kidney during the delayed surgery.

**Table 1:** Patients' clinical characteristics.

Clinical characteristics	*n*	%
Mean age (yr)	36.49 ± 15.207	
Male	36	80.0
Female	9	20.0
BMI (m/kg^2^)	24.85 ± 3.44	

Creatinine/(*μ*mol/L)		
Previous	67.32 ± 22.91	
Postoperation	62.84 ± 15.42	

BMI: body mass index.

**Table 2:** Injury position and type of Injury.

Type of injury	*n* (%)	Injury position	*n* (%)
Collision-related trauma	12 (26.7)	RK	7 (15.6)
		LK	5 (11.1)

Traffic accidents	27 (60.0)	RK	14 (31.1)
		LK	13 (28.9)

Falls	6 (13.3)	RK	3 (6.7)
		LK	3 (6.7)

RK: right kidney; LK: left kidney.

**Table 3:** Summary of operational characteristics.

Operational characteristics	*n* (%)
Delayed surgery	45 (100)
Preserved kidney success	44 (97.8)
Nephrectomy	1 (2.2)
Patients died	0

**Table 4:** Postoperative complications.

Adverse events	*n* (%)
Postoperative follow-up rate	35 (77.78, 35/45)
Hypertension	3 (8.6%, 3/35)
Microscopic hematuria	4 (11.4%, 4/35)
Urinary tract infection	2 (5.7%, 2/35)
Urinoma	2 (5.7%, 2/35)

## Data Availability

The analyzed data sets generated during the study are available from the corresponding author upon reasonable request.
